The article "Neurofibromatosis Type 1 and Diabetes Mellitus: An Unusual Association" was published in 2013. Journal: Case Rep Endocrinol.

# Neurofibromatosis Type 1 and Diabetes Mellitus: An Unusual Association

**DOI:** 10.1155/2013/689107

**Published:** 2013-10-29

**Authors:** Bayram Ozhan, Ali Aykan Ozguven, Betül Ersoy

**Affiliations:** ^1^Division of Pediatric Endocrinology and Metabolism, School of Medicine, Pamukkale University, Kınıklı, 20070 Denizli, Turkey; ^2^Division of Pediatric Oncology, School of Medicine, Celal Bayar University, 45020 Manisa, Turkey; ^3^Division of Pediatric Endocrinology and Metabolism, School of Medicine, Celal Bayar University, 45020 Manisa, Turkey

## Abstract

Neurofibromatosis type 1 is a multisystemic disease. It may manifest as abnormalities of the nervous tissue, bones, soft tissue, or skin. Autoimmune disease associated with NF1 can be seen. Diabetes mellitus is rarely seen in association with NF1. Here, we report a case with established NF1 who also had a diagnosis of diabetes mellitus.

## 1. Introduction

Neurofibromatosis type 1 (NF1) is one of the most common autosomal dominant conditions affecting ectodermal and mesodermal tissues, occurring with an estimated incidence of 1 in 2,500 to 3,000 individuals independent of ethnicity, race, and gender [1]. Von Recklinghausen described NF1 in detail in a case report published in 1882, but because of the varied presentation and pleiotropic nature of the disease, formal diagnostic criteria were established in 1987 and updated in 1997 by the National Institutes of Health Consensus Development Conference [2]. It is well known that patients with neurofibromatosis show an increased incidence of various neoplasms, most of these being tumors of neural crest origin including neurofibromas, leiomyomas, ganglioneuromas, paragangliomas, and carcinoids, but it has also been related to small bowel adenocarcinoma, pancreatic endocrine malignant tumor, and neurofibromatosis of the colon and urinary bladder.

Diabetes mellitus is rarely seen in association with NF1. Two children with diabetes mellitus associated with NF1 cases have been reported so far [3, 4]. Here, we report a case with established NF1 who also has a diagnosis with diabetes mellitus.

## 2. Case Report

A 9-year-old boy was admitted to the hospital with a history of polydipsia, polyuria, and enuresis nocturna for the last month. He was the first child of nonconsanguineous parents. His birth history was uneventful. His birth weight was 4000 gr (SDS: 0.95). His uncle has type 2 diabetes. On his physical examination, weight was 25 kg (SDS: 0.38), body mass index was 13,52 kg/m^2^ (SDS: 1.80), height was 136 cm (SDS: 1.42), blood pressure was 95/60 mmHg, and pulse rate was 95 bpm and rhythmic. His dermatological examination revealed multiple café-au-lait spots (>9) of 1–5 cm in diameter. He had two plexiform neurofibromas on his neck examination. Laboratory examination revealed a blood glucose level of 447 mg/dL; urinalysis revealed glucosuria and ketonuria; his blood ketone level was 2 mmol/L (normal level < 0.8). Acidosis was not detected on his concurrent blood gases analyses. Liver and renal functions were normal. Insulin level was <2 uU/mL (normal level 2.6–24.9), C-peptide level was 0.473 ng/mL (normal level 1.1–5), and HbA1c was 10.7% (normal range 4.6–6.4%). His thyroid function tests were normal. Islet cell antibodies (ICA) were 0.147 U/mL (normal range 0–1.1); insulin-associated antigen-2 antibody (IAA) was <0,032 (normal range < 0.4). His thyroid and celiac antibodies investigation was negative. The patient was diagnosed with neurofibromatosis type 1 and diabetes mellitus type 1. Insulin treatment was initiated, and normoglycemia was maintained on 0.8 units of insulin/kg/day. Later, the patient underwent further investigations to search for other characteristics of neurofibromatosis. Eye examination revealed no iris Lisch nodules. Osseous lesions were not detected on skeletal survey. Cranial magnetic resonance imaging (MRI) showed multiple hyperintense signal abnormalities in T2-weighted sequences. Abdominal ultrasonography and MRI were normal. Blood somatostatin level was 16 pg/mL (normal 0−26). On his regular followup, HbA1c level decreased to 6.9%.

## 3. Discussion

NF1, previously known as von Recklinghausen's disease, is a relatively common autosomal dominant disease [2]. The specific gene maps to chromosome 17q11.2. Clinical manifestations of NF1 include cafe-au-lait spots, freckling, generalized cutaneous neurofibroma, Lisch nodules, short stature, optic glioma, and CNS tumors. NF1 patients have increased risk of developing malignancies. They have a high spontaneous mutation rate, and mutations in tumor suppressor genes play an important role in the development of tumors [5]. The most common cause of death is CNS tumors.

There are few reports of NF1 patients associated with autoimmune diseases. The reported autoimmune diseases associated with NF1 are as follows: systemic lupus erythematosus, multiple sclerosis, membranous glomerulonephritis, IgA nephropathy, mixed connective tissue disease, juvenile arthritis, autoimmune hemolytic anemia, bullous pemphigoid, vitiligo, and autoimmune thyroiditis [2, 5].

Diabetes mellitus is rarely seen in association with NF1. It is attributed to the occurrence of somatostatinomas in the pancreas and the duodenum [3]. Somatostatinomas are rare endocrine tumors. They derive from the somatostatin-producing delta cells of the pancreas or the endocrine cells of the digestive tract and may be sporadic (93.1%) or familial (6.9%) in association with NF1, multiple endocrine neoplasia type 1 (MEN 1), and Von Hippel-Lindau syndrome [6]. The classic somatostatinoma syndrome, diabetes mellitus, diarrhea/steatorrhoea and cholelithiasis, typically occurs in pancreatic tumors, whereas duodenal tumors most often present with obstructive symptoms. These rare neoplasms have been reported only in adult and elderly patients. Since the clinical symptoms are often variable and nonspecific, great many somatostatinomas are “incidentalomas” found during cholecystectomy or in the course of gastrointestinal imaging studies. CT, MRI, selective arteriography of the celiac tripod, and endoscopic retrograde cholangiopancreatography are useful diagnostic tools for correctly locating the tumor [6]. Diagnosis may be confirmed by measuring the fasting plasmatic hormone concentration by means of the radioimmunoassay method. If the plasmatic basal levels of somatostatin do not indicate values that are at least three times the normal concentration, diagnostic tests, both stimulatory (with tolbutamide, calcium/pentagastrin, or secretin) and inhibitory (with diazoxide), can be performed.

Our patient was diagnosed with NF1 according to formal diagnostic criteria and diabetes mellitus type 1. He had multiple café-au-lait spots and two plexiform neurofibromas. Two or more clinical features signify the presence of NF1 in a patient [2]. We performed abdominal MRI and ultrasonography to detect any abnormality associated with NF1 and somatostatinoma. Although abdominal imaging was negative, we checked blood somatostatin level to exclude somatostatinoma. Somatostatin level was found within normal range. Two children with diabetes mellitus associated with NF1 cases have been reported. Zaka-ur-Rab and Chopra reported a 9-year-old-boy known to have NF1 since birth. He presented with polydipsia, polyuria, and polyphagia for the last 3 months. His blood glucose was 830 mg/dL. Urine examination showed specific gravity of 1.040, glucosuria of 4+, and traces of ketone bodies. The patient was put on insulin therapy, and normoglycemia was maintained on 0.8 units of insulin/kg. They had searched for somatostatinoma but did not mention anything about autoantibody against the pancreas. The second patient was reported by Kamoun et al. in 2009. The patient was a 15-year-old boy. He presented with polyuria, polydipsia, and weight loss of a few weeks' duration and vomiting with abdominal pain for the last 24 h. His family history was positive for NF1. His blood glucose level was 360 mg/dL, and he had a metabolic acidosis. Urine examination demonstrated glycosuria (4+) and ketonuria (3+). Following initial resuscitation, the patient commenced subcutaneous insulin, 0.8 units/kg/24 h. Glutamic acid decarboxylase (GAD) antibodies were positive (481 UI/mL, reference range <10 UI/mL). All the other autoantibodies, including insulin-associated antigen-2 antibody (IA-2), islet cell antibodies (ICA), antinuclear, antithyroid peroxidase, antithyroglobulin, and antiadrenal antibodies were undetectable.

Reported NF1 with diabetes patients, including our patient, were all male. This may be coincidental. One of the reported patients had GAD antibody, but the other did not. Our patient was searched for autoimmunity, but no positive antibody could be found. The pathological process causing diabetes mellitus is not yet clear. The NF1 gene is located on chromosome 17q11.2. Neurofibromin, the product of the nonmutated gene, has the activity of a GTPase-activating protein and is capable of downregulating the cellular p21-ras protooncogene. The loss of neurofibromin function may lead to uncontrolled cell growth or tumor formation, which may lead to increased tumor formation in patients with NF1 [7, 8]. Furthermore, abnormal neurofibromin production suppresses Fas ligand expression. This may prevent apoptosis of CD4+ T cells, which is important in the development of autoimmunity [1]. Decreased T cell apoptosis due to abnormal neurofibromin production may be an underlying factor for the development of the autoimmune diseases.

As the number of reports on the coexistence of NF1 and autoimmune diseases increases, an association rather than a coincidence becomes more likely.
